# Dual roles of miR-374a by modulated c-Jun respectively targets CCND1-inducing PI3K/AKT signal and PTEN-suppressing Wnt/β-catenin signaling in non-small-cell lung cancer

This article has been retracted.

**DOI:** 10.1038/s41419-017-0103-7

**Published:** 2018-01-23

**Authors:** Mengyang Zhao, Ping Xu, Zhen Liu, Yan Zhen, Yiyu Chen, Yiyi Liu, Qiaofen Fu, Xiaojie Deng, Zixi Liang, Yonghao Li, Xian Lin, Weiyi Fang

**Affiliations:** 1 Cancer Center, Integrated Hospital of Traditional, Chinese Medicine, Southern Medical University, Guangzhou, 510315 China; 2 Department of Oncology, The People’s Hospital of Zhengzhou University, Zhengzhou, Henan 450003 China; 3 Respiratory Department, Peking University Shenzhen Hospital, Shenzhen, 518034 China; 4 Key Laboratory of Protein Modification and Degradation, School of Basic Medical Sciences and Affiliated Cancer Hospital & Institute, Guangzhou Medical University, Guangzhou, 511436 China

## Abstract

MiR-374a appears to play a complex role in non-small-cell lung cancer (NSCLC). Here, we demonstrate a dual role for miR-374a in NSCLC pathogenesis. The effects and modulatory mechanisms of miR-374a on cell growth, migration, invasion, and in vivo tumorigenesis and metastasis in nude mice were also analyzed. The expression of miR-374a was examined in NSCLC and non-cancerous lung tissues by quantitative real-time reverse transcription-PCR (qRT-PCR), and in situ hybridization, respectively. miR-374a directly targets CCND1 and inactivates PI3K/AKT and Ras-mediated cell cycle signalings, as well as epithelial–mesenchymal transition (EMT). This not only dramatically suppressed cell growth, migration, invasion,and metastasis, but also elevated A549 and pc-9 NSCLC cell sensitivity to cisplatin (DDP) while increasing survival time of tumor-bearing mice. Interestingly, miR-374a serves an inverse function in SPCA-1 and H1975 NSCLC cells by directly targeting PTEN to activate Wnt/β-catenin and Ras signalings and its downstream cascade signals. Surprisingly, transcription factor c-Jun bound to the promoter region of human miR-374a and suppressed miR-374a in A549 and pc-9 cells while inducing it in SPCA-1 and H1975 cells. Increased levels of miR-374a appeared to serve a protective role by targeting CCND1 in early-stage NSCLC (Stages I and II). Inversely, increased miR-374a was an unfavorable factor when targeting PTEN in more advanced staged NSCLC patients. Our studies are the first to demonstrate that miR-374a plays divergent roles in NSCLC pathogenesis at different stages of the disease and implicate the potential application of miR-374a targeting for cancer therapy.

## Introduction

Lung cancer is one of the deadliest types of cancer as demonstrated by the poor survival and high relapse rates after surgery. Non-small-cell lung cancer (NSCLC) is the most commonly diagnosed type of lung cancer, and the 5-year survival rate is less than 15%^1^. Thus, further elucidating the molecular mechanisms of NSCLC is urgently required^2^.

Accumulating evidence has shown that microRNAs (miRNAs) play a pivotal role in NSCLC pathogenesis, which has provided new insights into targeted therapy of this disease^3–5^. Several studies have shown that miRNAs are frequently dysregulated in cancers and can modulate both oncogenes and tumor suppressor genes^6–10^. Among them, miR-374a has been frequently reported to be involved in the carcinogenesis and progression of many human malignancies. Expression of miR-374a was previously reported to be elevated in osteosarcoma cell lines and in colon cancer^11,12^. Furthermore, ectopic expression of miR-374a activated Wnt/β-catenin signaling to promote breast cancer epithelial-to-mesenchymal transition (EMT) and metastasis in vitro and in vivo by suppressing WIF1, PTEN, or WNT5A expression^13^. miR-374a promotes cell proliferation, migration, and invasion by targeting SRCIN1 in gastric cancer^14^. The above-mentioned studies suggest that miR-374a functions as an oncogene during cancer progression. However, in weakly invasive and metastatic breast cancer tumors, the relative expression of miR-374a was lower in the center than at the edges. An inverse relationship was noted for the highly invasive and metastatic group tumors, and miR-374a was lower in cancer tissues compared to normal tissues^15^.

In lung cancer, miR-374a was first reported to be upregulated in primary small cell lung cancer compared to normal lung^16^. Furthermore, functional assays revealed that miR-374a acts as an oncogene by directly targeting Wnt5a to regulate proliferation, gefitinib-induced apoptosis, EMT, migration, and invasion of NSCLC in vitro and in vivo^17^. Interestingly, low miR-374a expression in early-stage NSCLC was associated with poor patient survival^18^, which suggested that miR-374a may also serve a tumor-suppressive role in NSCLC. The latest research suggested that miR-374a suppresses lung adenocarcinoma cell proliferation and invasion by targeting TGFA gene expression^19^. Together, these data demonstrate a very paradoxical and inversed role of miR-347a in NSCLC. However, what are the real roles of miR-374a in NSCLC?

In this study, we found that human miR-374a inactivates the phosphatidylinositol-3-kinase (PI3K)/AKT and Ras pathways and directly suppresses expression of CCND1 which consequently inhibits A549 and pc-9 cell proliferation, EMT, and metastasis in vitro. miR-374a also enhanced A549 and pc-9 sensitivity to cisplatin (*cis*-Diammindichloroplatin (DDP)) *i*n vivo. miR-374a had the opposite effects in SPCA-1 and H1975 cells by targeting phosphatase and tensin homolog (PTEN) and activating the Wnt/β-catenin and Ras signaling pathway. Furthermore, we examined expression patterns of miR-374a in NSCLC by in situ hybridization and observed a correlation between miR-374a and CCND1 in early-stage NSCLC and a correlation between miR-374a and PTEN in the advanced NSCLC. Our studies are the first to demonstrate that miR-374a plays divergent roles in NSCLC pathogenesis at different stages of the disease and in different patients.

## Results

### miR-374a promotes SPCA-1 and H1975 cell proliferation, cell cycle transition, cell migration, invasion, and metastasis in vitro and in vivo

To understand the biological effects of miR-374a deregulation in human NSCLC cells, in vitro gain-of-function analyses were performed using lentivirus or mimics overexpression in A549, pc-9, SPCA-1, and H1975 cell lines (Supplementary Figure 1A). More than 10-fold increase in miR-374 expression was observed in miR-374a lentivirus or mimics-treated NSCLC cells compared with the control group by quantitative real-time reverse transcription-PCR (qRT-PCR) (with *P* < 0.01; *P* < 0.001) (Supplementary Figure 1B). To further explore its biological role in NSCLC, miR-374a inhibitors were transfected into Lv-miR-374a-A549 cells, Lv-miR-374a-pc-9 cells, Lv-miR-374a-SPCA-1, and Lv-miR-374a-H1975 cells, and expression levels of miR-374a were detected by qRT-PCR (Supplementary Figure 1C).

Subsequently, SPCA-1 and H1975 cell proliferation was measured in vitro. Compared with negative controls, we found that ectopic miR-374a promoted SPCA-1 and H1975 cell growth and G1 to S cell cycle transition by 3-(4,5-dimethylthiazol-2-yl)-2, 5-diphenyltetrazolium bromide (MTT) assay (Fig. 1a), colony formation assay (Fig. 1b), cell cycle analysis (Fig. 1c), and Edu assay (Fig. 1d, Supplementary Figure 1D). We also observed that miR-374a overexpression markedly promoted SPCA-1 and H1975 tumor growth (Fig. 1e and Supplementary Figure 1E).

**Fig. 1:** miR-374a promotes SPCA-1 and H1975 cell proliferation, migration, and invasion in vivo and in vitro The effect of miR-374a on the growth of SPCA-1 and H1975 NSCLC cells was examined by **a** MTT assay, **b** colony formation assay, **c** cell cycle analysis, and **d** EdU incorporation assay. Mean ± SD (*n* = 3). Scale bars, 100 μm. **e**. Excised tumors 20 days after implantation and representative, L (left) NC, R (right) miR-374a (*n* = 5). The effect of miR-374a on SPCA-1 and H1975 NSCLC cell migration and invasion was measured by **f** transwell assay and **g** Boyden Chamber assays. Mean ± SD (*n* = 3). Scale bars, 100 μm. **h** Representative bioluminescence imaging of the lungs. On day 30, mice receiving transplants of indicated cells were killed and lungs were collected. **i** Lung metastases were confimed by H&E staining. Scale bars, 200 μm. Arrows indicate nests of malignant cells. Mean ± SD (*n* = 3). *P < 0.05

To examine the effects of miR-374a overexpression on migration and invasion, Lv-miR-374a cells were cultured with or without inhibitors. Compared with LEV control cells, we found that miR-374a significantly promoted cell migration and invasion in transwell and Boyden Chamber assays. The addition of inhibitors could rescue this effect in SPCA-1 and H1975 cells (Fig. 1f, g, and Supplementary Figure 1F and G).

Since in vitro experiments revealed that miR-374a expression was associated with metastatic phenotypes, we next asked whether this effect was present in vivo. SPCA-1 and H1975 cells stably expressing miR-374a were transplanted under the liver capsule of mice and tissues were harvested 4 weeks later and the result showed that mice bearing SPCA-1/miR-374a and H1975/miR-374a tumors developed prominent lung metastases (Fig. 1h, i). Histological analyses further revealed that miR-374a could promote metastasis of SPCA-1 and H1975 cells (Supplementary Figure 1H). Together, these data indicate that miR-374a as a potential oncogene promotes cell proliferation, migration, and invasion in SPCA-1 and H1975 cell lines.

### miR-374a inhibits A549 and pc-9 cell proliferation, cell cycle transition, cell migration, invasion, and metastasis in vitro and in vivo

Subsequently, A549 and pc-9 cell proliferation was measured in vitro. Compared with negative controls, we interestingly found that ectopic miR-374a inhibited A549 and pc-9 cell growth and G1 to S cell cycle transition by MTT assay (Fig. 2a), colony formation assay (Fig. 2b, Supplementary Figure 2A), cell cycle analysis (Fig. 2c), and Edu assay (Fig. 2d, Supplementary Figure 2B). We also observed that miR-374a overexpression markedly suppressed *i*n vivo tumorigenesis of A549 and pc-9 cells tumor growth (Fig. 2e, Supplementary Figure 2C). These above-mentioned results indicated that miR-374a could inhibit cell proliferation in A549 and pc-9 cells.

**Fig. 2:** miR-374a reduces A549 and pc-9 cell proliferation, migration, and invasion in vivo and in vitro The effect of miR-374a on the growth of A549 and pc-9 cells was examined by **a** MTT assay, **b** cell cycle analysis, **c** colony formation assay, and **d** EdU incorporation assay. Mean ± SD (*n* = 3). Scale bars, 100 μm. Excised tumors 20 days after implantation. L (left) NC, R (right) miR-374a (*n* = 5). **e**, **f** The effect of miR-374a on A549 and pc-9 cell migration and invasion was measured by transwell assay and Boyden Chamber assays. Mean ± SD (*n* = 3). Scale bars, 100 μm. **g** Representative bioluminescence imaging of the lungs. On day 30, mice receiving transplants of indicated cells were killed and lungs were collected and lung metastases were confimed by H&E staining. Scale bars, 200 μm. Arrows indicate nests of malignant cells. Mean ± SD (*n* = 3). *P < 0.05

To examine the effects of miR-374a overexpression on migration and invasion, Lv-miR-374a cells were cultured with or without inhibitors. Compared with LEV control cells, we found that miR-374a significantly reduced cell migration and invasion in transwell and Boyden Chamber assays. The addition of inhibitors could rescue this effect in A549 and pc-9 cells (Fig. 2f).

Since in vitro experiments revealed that miR-374a expression was associated with metastatic phenotypes, we next asked whether this effect was presented in vivo. A549 and pc-9 cells stably expressing miR-374a were transplanted under the liver capsule of mice and tissues were harvested 4 weeks later. Strikingly, mice bearing A549/LEV and pc-9/LEV tumors developed prominent lung metastases, whereas no visible metastases were found in mice transplanted with A549/miR-374a and pc-9/miR-374a cells (Fig. 2g). Histological analyses further revealed that miR-374a could inhibit A549 and pc-9 metastasis. Together, these data indicate that miR-374a plays a pivotal role in NSCLC metastasis in vitro and in vivo but its function is unique in different NSCLC cell lines.

### miR-374a directly targets CCND1 3′UTR in A549 and pc-9 and PTEN 3′UTR in SPCA-1 and H1975 cells

To delineate the mechanism by which miR-374a inhibited or promoted cell proliferation, invasion, and migration in NSCLC cells, we used TargetScan (http://www.targetscan.org/) and PicTar (http://pictar.mdc-berlin.de/) bioinformatics algorithms. We found that CCND1 and PTEN were predicted to be direct targets of miR-374a (Fig. 3a). Western blot analysis revealed that miR-374a mimics downregulated CCND1 expression in A549 and pc-9 and PTEN in SPCA-1 and H1975 cells, respectively (Fig. 3b). Conversely, transfection of miR-374a inhibitors into these four lines resulted in upregulation of CCND1 or PTEN (Fig. 3b). No significant change in PTEN protein was observed for A549-miR-374a and pc-9-miR-374a cells but CCND1 was upregulated in SPCA-1-miR-374a and H1975-miR-374a cells (Fig. 3c). We next performed luciferase reporter assays to validate that miR-374a could directly target the 3′-untranslated region (UTR) of CCND1 and PTEN in NSCLC cells. We found that miR-374a could directly target the CCND1 3′UTR (Fig. 3d) but not the PTEN 3′UTR in A549 and pc-9 cells (Supplementary Figure 3A, 3B). In SPCA-1 and H1975 cells, miR-374a directly targeted the PTEN 3′UTR (Fig. 3d) but not the CCND1 3′UTR (Supplementary Figure 3B, 3C). Immunohistochemistry of xenografts derived from A549-miR-374a, pc-9-miR-374a, SPCA-1-miR-374a, or H1975-miR-374a cells revealed a drastic reduction in CCND1 and PTEN expression, respectively (Fig. 3e). Taken together, these data suggest that miR-374a directly suppresses CCND1 in A549 and pc-9 cells but PTEN in SPCA-1 and H1975 cells.

**Fig. 3:** miR-374a directly regulates CCND1 in A549 and pc-9 cells or PTEN in SPCA-1 and H1975 respectively **a** miR-374a and its putative binding sequences in the 3′UTRs of CCND1 and PTEN. Mutations were generated in the complementary site that binds to miR-374a. **b**,** c**. Western blotting detected protein levels of CCND1 and PTEN in miR-374a-overexpressing or miR-374a-inhibited NSCLC cells, with β-actin serving as a loading control. **d** Luciferase reporter assays were used to determine whether miR-374a directly targets the 3′UTR of CCND1 in A549 and pc-9 cells and PTEN in SPCA-1 and H1975 cells. Mean ± SD (*n* = 3). *P < 0.05. **e** Expression of CCND1 and PTEN was evaluated using immunohistochemistry of NSCLC xenografts. Scale bars, 50 μm. **f** Protein levels of CCND1, p-PI3K, p-AKT, E-cadherin, N-cadherin, c-MYC, CDK4, and P21 were detected by western blot in A549 and pc-9 cells after transfection with NC or CCND1 siRNA. **g** Protein levels of PTEN, β-catenin, TCF4, N-cadherin, c-MYC, and P21 were detected by western blot in SPCA-1 and H1975 cells after transfection with NC or PTEN siRNA

Levels of p-PI3K, p-AKT, c-Myc, CDK4, and N-cadherin were significantly reduced while E-cadherin and P21 were increased after small-interfering RNA (siRNA)-mediated suppression of CCND1 in A549 and pc-9 cells (Fig. 3f). Downregulation of PTEN in SPCA-1 and H1975 cells increased the expression of invasion-associated genes including β-catenin, TCF4, and N-cadherin, as well as elevated oncogenic cell cycle regulator c-Myc but reduced P21 (Fig. 3g). These results indicate that miR-374a can mediate CCND1 and PTEN and their downstream factors.

### Ectopic expression of CCND1 or PTEN mitigates miR-374a-mediated effects on proliferation, invasion, and migration in NSCLC cells

To explore whether miR-374a targeting of CCND1 or PTEN was responsible for its effects on proliferation, migration, and invasion, we utilized an expression construct that encodes the entire CCND1 and PTEN coding sequence but lacks the 3′UTR. These functional studies demonstrated that CCND1 or PTEN overexpression respectively inhibited or promoted proliferation, migration, and invasion (Fig. 4a–c and Supplementary Figure 4A, 4B). Ectopic expression of CCND1 or PTEN partially rescued miR-374a-mediated effects on growth, migration, and invasion in A549 and pc-9 or SPCA-1 and H1975 cells, respectively (Fig. 4a–c and Supplementary Figure 4A, 4B). This suggested that the effects of miR-374a overexpression in NSCLC cells specifically depend on CCND1 or PTEN suppression.

**Fig. 4:** Ectopic expression of CCND1 or PTEN attenuates miR-374a-mediated effects on proliferation, invasion, and migration in A549, pc-9, SPCA-1, and H1975 cells **a** EdU incorporation assays, **b**,** d** transwell migration assays and Boyden Chamber assays for A549, pc-9, SPCA-1, and H1975 cells were performed after transfection with NC, ectopic CCND1, PTEN, and/or miR-374a as indicated. Mean ± SD (*n* = 3). Scale bars, 100 μm. *P < 0.05. **d** miR-374a modulates expression of cell cycle-associated and EMT-related genes via inactivating PI3K/AKT and Ras pathways in A549 and pc-9 cells or activating β-catenin and Ras signalings in SPCA-1 and H1975 cells. Cell cycle regulators, including c-MYC, P21, CCND1, and CDK4, and invasion-marker genes, including ZEB2, TCF4, β-catenin, E-cadherin, and N-cadherin, were detected after transfection with NC, ectopic CCND1, PTEN, miR-374a, and/or inhibitors as indicated in NSCLC cells by western blot

### miR-374a modulates expression of cell cycle-associated and EMT-related genes by inactivating PI3K/Akt and Ras signalings or activating β-catenin and Ras signalings

To explore the molecular mechanisms by which miR-374a mediates its effects through CCND1 or PTEN, we examined protein levels of several cell cycle and invasion-associated genes in Lv-miR-374a cells transfected with ectopic CCND1 or Lv-miR-374a inhibitor-treated cells after PTEN overexpression. As shown in Fig. 4d, we observed that miR-374a not only suppressed levels of phos-PI3K (Tyr458), phos-Akt (Ser473), K-Ras, and p-Erk, but also significantly decreased the expression of cell cycle-related genes including CCND1, c-Myc, and CDK4 in A549 and pc-9 cells. Mesenchymal marker N-cadherin was also downregulated while E-cadherin expression was increased. Overexpression of miR-374a in SPCA-1 and H1975 cells increased the expression of β-catenin, TCF4, K-Ras, p-Erk, ZEB2 and N-cadherin, CCND1, and c-Myc but decreased P21 (Fig. 4e). Suppressing miR-374a with specific inhibitors or by overexpressing CCND1 or PTEN both reversed effects mediated by ectopic miR-374a (Fig. 4d, e). Taken together, these data suggest that in A549 and pc-9 cells, miR-374a suppresses cell growth and metastasis by inactivating the PI3K/Akt and Ras pathways, thus modulating its downstream cell cycle and EMT-related genes. However, in SPCA-1 and H1975 cells, miR-374a exerts its effects by activating β-catenin and Ras signalings, consistent with a previous report of miR-374a function in breast cancer^13^.

### c-JUN binds the promoter region of human miR-374a

We used siRNAs to suppress c-JUN expression of A549 and pc-9, SPCA-1, and H1975 cells (Fig. 5aa). Subsequent qPCR analysis indicated that the expression of miR-374a was markedly increased in A549 and pc-9 cells but decreased in SPCA-1 and H1975 cells (Fig. 5ab). Further, bioinformatics predictions (UCSC, PROMO, and GeneCards) indicated that the promoter region of human miR-374a contains two c-JUN binding sites (Fig. 5b). Using chromatin immunoprecipitation (ChIP), we confirmed that c-JUN could bind the putative miR-374a promoter in A549 and pc-9, SPCA-1 and H1975 cells (Fig. 5c). Furthermore, a reduction in the wild-type miR-374a promoter luciferase activity was observed upon upregulation of c-JUN in the A549 and pc-9 cells and a similar effect was observed when either site A or site B were individually mutated (*P* < 0.05). However, c-JUN overexpression did not result in a further reduction of luciferase activity when both sites A and B were mutated (Fig. 5d). Conversely, ectopic c-JUN expression activated the transcription of firefly luciferase by driving the wild-type miR-374a promoter in SPCA-1 and H1975 cells. When the binding sequence of site A was mutated, firefly luciferase expression dropped 2.5-fold in SPCA-1 and 2.2-fold in H1975 cells. When the binding sequence of site B was mutated, firefly luciferase expression dropped 2.7-fold in SPCA-1 and 2.6-fold in H1975 cells (Fig. 5d). These data indicate that c-JUN binds to the promoter of miR-374a and inhibits its transcription in A549 and pc-9 cells but promotes transcription in SPCA-1 and H1975 cells. Taken together, c-JUN is involved in miR-374a transcription, and two c-JUN binding sites in the miR-374a promoter are functional in A549 and pc-9 cells, SPCA-1, and H1975 cells.

**Fig. 5:** c-JUN binds the promoter region of human miR-374a that mediates its effects on cell proliferation, migration, and invasion in A549, pc-9, SPCA-1 and H1975 cells **a** (a) siRNAs were used to suppress c-JUN expression as shown by qPCR. **a** (b) Knocking down c-JUN respectively stimulated or inhibited expression of miR-374a in NSCLC cells. **b** Schematic representation of the promoter regions of miR-374a with putative c-JUN TFBSs (**a**, **b**) and the structure of the wild-type (WT) and TFBS mutant (MutA, MutB, and MutAB) luciferase reporters driven by the promoter. **c** ChIP assay using antibodies against c-JUN in NSCLC cells; PCR gel showing amplification of c-JUN-binding sites A and B. **d** Relative luciferase activity of the indicated promoter vectors in A549, pc-9, SPCA-1, or H1975 cells transfected with c-JUN plasmids. **e** EdU incorporation assays, **f** transwell migration assays, and **g** Boyden Chamber invasion assays of NSCLC cells were performed after transfection with NC, c-JUN siRNA, miR-374a mimics and/or inhibitors as indicated. Mean ± SD (*n* = 3). Scale bars, 100 μm. *P < 0.05. **h** Protein levels of CCND1 and PTEN were detected by western blot in NSCLC cells after transfection with NC, c-JUN siRNA, miR-374a mimics, and/or inhibitors

### miR-374a restores the effects on cell proliferation, migration, and invasion induced after c-JUN suppression in NSCLC cells

To explore whether c-JUN binding to the promoter region of human miR-374a was responsible for its effects in NSCLC cells, we transfected miR-374a inhibitors or mimics respectively into si-JUN A549, pc-9, SPCA-1, or H1975 cells. Proliferation (Fig. 5e, Supplementary Figure 5A), migration (Fig. 5f, Supplementary Figure 5B), and invasion (Fig. 5g, Supplementary Figure 5B) were significantly increased in si-JUN A549 and pc-9 cells treated with miR-374a-inhibitors or si-JUN SPCA-1 and H1975 cells treated with miR-374a-mimics. Western blot analysis confirmed that c-JUN could regulate miR-374a and its direct targets CCND1 in A549 and pc-9 or PTEN in SPCA-1 and H1975 cells (Fig. 5h).

### Clinical significance of miR-374a in NSCLC

PCR analysis indicated that miR-374a expression levels were significantly increased in NSCLC samples compared to paracancerous tissue (PT) (*P* = 0.0014) (Fig. 6a). Expression of miR-374a was significantly overexpressed in NSCLC tissues compared with PT (Fig. 6b). miR-374a was highly expressed in 72.2% (114/158) of NSCLC samples, while only in 37.3% (59/158) of PT samples, a significantly lower frequency (*P* = 0.000) (Supplementary Table 1). Clinical characteristics of the NSCLC patients have been summarized in the Supplementary Table 2. We did not find a significant association between miR-374a expression level and patient age, sex, FIGO (International Federation of Gynecology and Obstetrics) stage (I–II vs. III–IV), tumor size (T classification), or distant metastasis stage (M classification) in the 158 NSCLC cases. However, we observed that the expression level of miR-374a was positively correlated with lymph node status (N classification; N0–N1 vs. N2–N3) (*P* = 0.040) (Supplementary Table 2). Subsequently, univariate analyses showed that age (*P = *0.005), N classification (*P < *0.001), FIGO stage (*P = *0.007), and miR-374a expression (*P = *0.041) were significantly correlated with patient survival (Supplementary Table 3). To determine whether miR-374a expression level is an independent prognostic factor for NSCLC, we performed multivariate analysis of miR-374a expression levels adjusted for age, N classification, and FIGO stage. These results showed that the level of miR-374a expression was not an independent prognostic factor (*P = *0.221) (Supplementary Table 3). Finally, we found that NSCLC patients with low miR-374a expression had longer survival compared with patients with high miR-374a levels (*P = *0.037, Fig. 6c). Interestingly, we found that low expression of miR-374a in early-stage NSCLC is associated with poor patient survival (*P = *0.046, Fig. 6d), which was consistent with a previous report of miR-374a in NSCLC^17^. Furthermore, in patients with advanced NSCLC, low levels of miR-374a correlated with longer survival (*P = *0.000, Fig. 6e). These results provide support that miR-374a plays distinct roles at different stages of NSCLC tumorigenesis.

**Fig. 6:** miR-374a expression in NSCLC is associated with poor prognosis and its relationship with CCND1 expression **a** Compared with paracancerous tissue (PT), miR-374a expression was markedly increased in NSCLC tissues (*P* = 0.0014). **b** miR-374a expression was examined in NSCLC and control tissues (Scale bars, 50 μm). (**a**,** b**) Positive expression of miR-374a in NSCLC tissues. **c** Negative miR-374a expression in NSCLC tissues. **d**. Negative miR-374a expression in PT. **c**. Kaplan–Meier survival analysis of overall survival for 158 NSCLC patients. **d**. Kaplan–Meier survival analysis in 81 early stage (Stage I or II) NSCLC specimens. **e** Kaplan–Meier survival analysis in 77 Stage II–IV NSCLC specimens. **f**,** h** Expression of miR-374a is associated with CCND1 and PTEN levels in NSCLC specimens. Three representative cases are shown. Scale bars, 200 μm and 50 μm, respectively. **g** Percentage of early-stage NSCLC specimens exhibiting low or high miR-374a expression in relation to CCND1 expression. **i** Percentage of advanced-stage NSCLC specimens exhibiting low or high miR-374a expression in relation to PTEN expression. **j** Patients with both high miR-374a expression and low CCND1 expression group had longer survival times only in early-stage NSCLC (*P* < 0.001). **k** Patients with low miR-374a expression and high PTEN expression group had longer survival times only in advanced-stage NSCLC (*P* < 0.001)

### Clinical association between miR-374a and CCND1 or miR-374a and PTEN expression in NSCLC specimens

We next asked whether there was an association between the expression level of miR-374a and CCND1 in NSCLC tissues. Unfortunately, we did not find a significant association between miR-374a and CCND1 expression in the whole NSCLC cohort (Supplementary Figure 5A) (*P* = 0.1550) nor only advanced NSCLC specimens (Stages III and IV) (Supplementary Figure 5B) (*P* = 0.8720). However, as shown in Fig. 6g, 81% of samples with low CCND1 expression exhibited high levels of miR-374a (22/27 cases), whereas 35% of samples with high CCND1 expression had low expression of miR-374a (19/54 cases) in early stage of NSCLC specimens (Stages I–II) (*P = *0.0164). More interestingly, as shown in Fig. 6i, 80% of samples with low PTEN expression exhibited high levels of miR-374a (39/49 cases), whereas 36% of samples with high PTEN expression had low expression of miR-374a (10/28 cases) in advanced NSCLC specimens (Stages III and IV) (*P = *0.0117). There was no correlation between miR-374a and PTEN levels in our whole NSCLC cohort (Supplementary Figure 6C) (*P* = 0.3920) nor only early stage of NSCLC specimens (Stages I–II) (Supplementary Figure 6D) (*P* = 0.0922). In early-stage NSCLC, patients with high miR-374a expression together with low CCND1 expression groups had significantly longer survival times (Fig. 6j) (*P* < 0.001). This effect was not observed for patients with advanced-stage NSCLC (Supplementary Figure 5E) (*P* = 0.475) nor the entire NSCLC cohort (Supplementary Figure 6F) (*P* = 0.088). Patients with low miR-374a expression together with high PTEN expression had the longest survival times among advanced-stage patients (Fig. 6k) (P < 0.001) as well was the entire NSCLC cohort (Supplementary Figure 6H) (*P* = 0.005). This effect was not found for early-stage NSCLC patients (Supplementary Figure 6G) (*P* = 0.916).

### miR-374a affects NSCLC cell chemosensitivity to DDP via respective downregulation of CCND1 or PTEN

Stably overexpressing miR-374a significantly sensitized A549 and pc-9 cells to DDP while SPCA-1 and H1975 cells become more resistant to this treatment. Inhibition rates induced 48 h after treatment with different concentrations of DDP were calculated for NSCLC cells before and after miR-374a transfection, and a fitted curve was used to calculate half-maximal inhibitory concentration (IC_50_) (Supplementary Figure 7A). The IC_50_ for DDP in A549 and pc-9 cells was decreased from 6.5 µM and 5.7 µM to 1.5 µM and 2.0 µM after miR-374a transfection. Conversely, the IC_50_ for SPCA-1 and H1975 cells increased from 2.4 µM and 3.0 µM to 8.4 µM and 7.8 µM respectively following transfection with miR-374a. Furthermore, we found that overexpression of CCND1 or PTEN significantly reversed the effects on DDP sensitivity induced by miR-374a overexpression (Supplementary Figure 7A).

We further evaluated the in vivo efficacy of DDP in mice bearing tumors originating from cells overexpressing miR-374a. To investigate the prognostic value of miR-374a expression in NSCLC, we evaluated its association with mouse survival using Kaplan–Meier analysis with the log-rank test. Among 36 mice bearing abdominal cavity tumors, we observed that DDP significantly increased survival time, and this effect was considerably more pronounced for the miR-374a overexpression group (Supplementary Figure 7B) (*P* < 0.01). Interestingly, the opposite results were observed in parallel groups using SPCA-1 cells to initiate tumors (Supplementary Figure 7B).

## Discussion

Accumulating evidence has demonstrated that aberrant expression of miRNAs is related to tumorigenesis, progression, and prognosis of various types of human cancers including NSCLC^20–22^. miR-374a, located on chromosome Xq13.2, seems to play dual roles in promoting or limiting the development of lung cancer according to several studies^16–18^. Here, we validated the phenotype induced by miR-374a but also explored the molecular mechanisms by which it exerts its effects.

In order to evaluate its function in NSCLC, miR-374a overexpression was found to markedly suppress proliferation, invasion, and metastasis of A549 and pc-9 cells in vitro and in vivo. These findings suggested that miR-374a functions as a tumor-suppressor in this line. Conversely, miR-374a serves an oncogenic role in the SPCA-1 and H1975 cell lines. Cisplatin (DDP)-based chemotherapy is still the standard first-line treatment for NSCLC, but chemoresistance limits its clinical efficacy^23^. We observed that ectopic miR-374a dramatically sensitized A549 and pc-9 cells to DDP as well as increased survival time of tumor-bearing mice. In contrast, miR-374a overexpression reduced SPCA-1 and H1975 cell sensitivity to DDP. Together, these data suggest that miR-374a exerts divergent effects in different NSCLC cells, likely due to intrinsic characteristics of cell lines.

Molecular mechanisms underlying the proliferation, invasion, metastasis, and chemotherapy resistance of NSCLC have been intensively studied. Cellular signaling pathways, such as Wnt/β-catenin and PI3K/Akt and Ras and their downstream signals including cell cycle and EMT, have been found to be aberrantly activated and play vital roles in the carcinogenesis and chemotherapeutic resistance^24–29^. In a previous study, miR-374a was able to constitutively activate Wnt/β-catenin signaling in breast cancer cells^13^. Thus, by suppressing WIF1, PTEN, or WNT5A, miR-374a may serve as an anti-metastasis therapeutic target in breast cancer. Consistent with this evidence, we found that in SPCA-1 and H1975 cells, miR-374a targets PTEN and further stimulates the Wnt/β-catenin pathway and its downstream cell cycle and EMT signals including inducing β-catenin, TCF4, ZEB2, N-cadherin, c-Myc, and CCND1, while decreasing P21. This result supports that miR-374a can serve as an oncogene in NSCLC. Interestingly, in A549 and pc-9 cells, miR-374a was observed to directly target the CCND1 oncogene, but not PTEN, which further inactivated PI3K/AKT and its downstream cell cycle and EMT signals. This included decreasing the expression of cell cycle-related genes such as c-Myc, CDK4, and mesenchymal marker N-cadherin, while increasing the expression of E-cadherin. What’s more, miR-374a could also activate Ras signal in SPCA-1 and H1975 cells and inactivate Ras signal in A549 and pc-9 cells. These demonstrated that miR-374a is a potential tumor suppressor in A549 and pc-9 cells, which was consistent with our study in colon cancer^30^ and nasopharyngeal carcinoma^31^ and the investigation of Wu et al.^19^. Overall, miR-374a plays a dual role through respectively targeting different genes and their downstream pathways, which underscores a complex role for miR-374a in NSCLC pathogenesis.

In previous study, c-Jun was found to suppress the expression of miR-374a^32^. In this study, we observed that c-JUN negatively regulated miR-374a expression in A549 and pc-9 cells, consistent with a previously published report^32^. However, inversed data indicated that c-JUN induces miR-374a expression in SPCA-1 and H1975 cells, which demonstrated a complex modulation mechanism for c-JUN-mediated regulation of miR-374a in NSCLC. c-JUN is an oncogenic transcription factor known to be an essential regulator of major biological events^33–35^. However, there were no reports demonstrating that c-JUN as a key oncongenic transcription factor binds to the promoter of miR-374a. Furthermore, ChIP assay confirmed c-JUN could bind to the promoter of miR-374a in A549, pc-9, SPCA-1, and H1975 cells. Furthermore, luciferase assays showed that c-JUN inhibits miR-374a transcription in A549 and pc-9 cells but promotes miR-374a transcription in SPCA-1 and H1975 cells. Together, these data confirm that miR-374a is directly modulated by c-JUN and serves distinct roles in different NSCLC cell lines.

miRNAs have been reported to play different roles depending on the tumor type. Dysregulation of miR-184 promotes cell proliferation in hepatocellular carcinoma by targeting INPPL1 and SOX7^36,37^. In addition, miR-184 acts as a tumor suppressor in nasopharyngeal carcinoma, lung cancer, and neuroblastoma by targeting c-Myc, BCL-2, and AKT2^38–40^. Aberrant miR-9 levels have been reported in many types of cancer, suggesting that miR-9 is involved in tumor pathogenesis. However, by modulating various mRNA targets, miR-9 may have opposing effects on proliferation in different types of cancer cells^41–44^. The functional divergence for the same miRNA in different tumor types is most likely attributed to distinct target genes. Consistent with this notion, we observed that miR-374a serves dual roles in different NSCLC cells.

Previously, Miko et al.^16^ reported that miR-374a is upregulated in primary small cell lung cancer. High expression of miR-374a was also associated with poor disease-free survival in NSCLC^17^. These two studies supported miR-374a as a potential oncogene promoting lung cancer progression. Consistent with their results, our findings showed that miR-374a expression levels were significantly increased in NSCLC samples and positively linked to N classification. Inversely, Wu et al.^19^ found the expression of miR-374a was downregulated in NSCLC which was based on the database of Cancer Genome Atlas. The differences of the results between the data of Wu et al.^19^ and our data may be due to the different sample sources or miR-374a data from the Cancer Genome Atlas microarray lacking the validation by qPCR. Interestingly, we observed that low expression of miR-374a in early-stage NSCLC was associated with poor patient survival. These data were consistent with the investigation of Vosa et al.^18^ and thus suggested that miR-374a functioned as a tumor suppressor in early-stage NSCLC. The discrepancy between the role of miR-374a early stage or advanced is similar to that of transforming growth factor-β (TGFβ)^45^. TGFβ is able to suppress growth in normal epithelial cells and during the early stages of tumorigenesis. However, upon accumulation of genetic and epigenetic alterations in tumor cells, it promotes an invasive and metastatic phenotype, accompanied by a progressive increase in secreted TGFβ levels. Unfortunately, although we observed that miR-374a expression was significantly correlated with patient survival based on the univariate analysis, it was not an independent prognosis factor through multivariate analysis. These present data may be mostly due to insufficient sample number detection or the complicated roles of miR-374a. Furthermore, we found that miR-374a expression correlated with CCND1 only in early-stage NSCLC tissues. Conversely, miR-374a expression was related to PTEN only in advanced NSCLC tissues. High miR-374a together with low CCND1 prolonged survival times but only for early-stage NSCLC patients. In contrast, advanced-stage NSCLC patients with the combination of low miR-374a expression and high PTEN expression had longer survival times. These data suggest that miR-374a plays a protective role in the early NSCLC by targeting CCND1 and acts as an oncogene at advanced stages by targeting PTEN.

Together, these results demonstrated that miR-374a acts as a double-edge sword during carcinogenesis and tumor progression of NSCLC. MiR-374a functions as a tumor suppressor early in the carcinogenic process but switches to a pro-oncogenic agent in late-stage disease. At this late stage, loss of miR-374a response actually prevents further progression by suppressing certain tumor suppressor, such as PTEN. This result represents a valuable resource to mine for information about the mechanisms that underlie the opposing roles of miR-374a at different stages in NSCLC progression and the changes in molecular and biological context that cause miR-374a to switch from tumor suppressor to tumor promoter in late-stage disease.

Although the underlying mechanisms leading to different effects of miR-374a remain to be investigated, it is possible that the role of miR-374a in tumorigenesis is highly dependent on the cell type and clinical stages of tumor development. However, since miR-374a exerts complex functions acting both as a tumor suppressor and a tumor promoter, inhibition of miR-374a as a therapeutic strategy must be approached with caution. The future use of miR-374a modulating drugs in the clinic must be carefully assessed, considering their effects on early-stage NSCLC tissues and advanced stages.

## Materials and methods

### Cell culture and tissue specimens

A549 cells were cultured in Dulbecco’s modified Eagle’s medium (DMEM, HyClone, Logan, UT) supplemented with 10% fetal bovine serum (FBS) (ExCell, Shanghai, China); pc-9, SPCA-1, and H1975 cells were cultured in RPMI-1640 medium (HyClone, Logan, UT) supplemented with 10% FBS (ExCell, Shanghai, China). Both cell lines were incubated in a humidified chamber with 5% CO_2_ at 37 °C. A tissue microarray with 158 NSCLC samples and 158 PT samples was purchased from Shanghai Outdo Biotech Co., Ltd China.

### RNA isolation, reverse transcription, and qRT-PCR

RNA was extracted from the NSCLC cell lines, tissues, and paracancerous tissue by Trizol (Takara Bio, Inc., Shiga, Japan). ARF5 and U6 genes were used as gene and miRNA internal controls, respectively. Cycling conditions were 95 °C for 10 min to activate DNA polymerase, followed by 45 cycles of 95 °C for 15 s, 60 °C (for miR-374a, c-JUN) for 15 s, and 72 °C for 10 s. Specificity of amplification products was confirmed by melting curve analysis. Independent experiments were done in triplicate. Specific sense primers of miR-374a, C-JUN, U6, and ARF5 are shown in Supplementary Table 4.

### Lentivirus production and infection

Lentiviral particles carrying hsa-miR-374a precursor and its flanking control sequence (NC for short) were constructed by GeneChem, Shanghai, China. A549, pc-9, SPCA-1, and H1975 cells were infected with lentiviral vector and polyclonal cells with green fluorescent protein signals were selected for further experiments using fluorescence-activated cell sorting flow cytometry. Total RNA from these cell clones was isolated, and levels of miR-374a were quantified using qRT-PCR.

### In situ hybridization

In situ hybridization was performed on formalin-fixed, paraffin-embedded sections (4 μm thickness) of tumor specimens. After processing with 3% H_2_O_2_, sections were treated with proteinase K (2 μg/ml) at 37 °C for 30 min, washed, and prehybridized for 2 h at 37 °C. Hybridization with digoxygenin (DIG)-labeled miRCURY LNA probes (probe sense: 5′-cACTTATCAGGTTGTATTATAa -3′; Biosense Bioscience Co., Ltd, Guangzhou, China) was performed overnight at 37 °C. Slides were then washed at 37 °C and incubated with alkaline phosphatase–conjugated sheep anti-DIG Fab fragments for 1 h at room temperature. Staining was visualized by adding BM purple AP substrate (Roche, Basel, Switzerland) according to the manufacturer’s instructions.

### Transient transfection with siRNAs, plasmid, or miR-374a mimics/inhibitors

The siRNAs for c-JUN, PTEN, CCND1, or miR-374a mimics and its inhibitors were designed and synthesized by RiboBio Inc. (Guangzhou, China). The sequence of the c-JUN, PTEN, CCND1 siRNAs, or miR-374a mimics and its inhibitors and their controls are shown in Supplementary Table 5. CCND1, PTEN, and c-JUN plasmids were purchased from Biosense (Guangzhou, China). At 24 h before transfection, A549, pc-9, SPCA-1, or H1975 NSCLC cells were seeded onto a 6- or 96-well plate (Nest, Biotech, China) at 30–50% confluence. The siRNA and plasmid of CCND1 and PTEN and miRNAs were then transfected at a working concentration of 100 nM using TurboFect siRNA Transfection Reagent (Fermentas, Vilnius, Lithuania) according to the manufacturer’s protocol. Cells were collected after 48–72 h.

### Western blotting analysis

Western blotting analysis was performed according to a previous description^46^. Antibodies included anti-PTEN, CDK1, p21, β-catenin, N-cadherin, E-cadherin, TCF4, c-Myc, c-JUN, AKT, p-AKT (Ser473), PI3K, p-PI3K (Tyr458), Ras, p-ERK, and p27 antibodies (1:1000; Cell Signaling Technology, Danvers, MA, USA) and ZEB2, CDK4, and β-actin antibody (1:500; Santa Cruz Biotechnology). Images were captured with ChemiDocTM CRS+Molecular Imager (Bio-Rad).

### Cell proliferation and cytotoxicity analyses

The MTT assay was used to examine cell viability. NSCLC cells (1000/well) were seeded in 96-well plates. For lentivirus-mediated miR-374a overexpression, the cells were incubated for 1, 2, 3, 4, 5, 6, or 7 days. For transient transfection with miR-374a mimics and miR-374a inhibitor, the cells were cultured for 1, 2, 3, or 4 days. Subsequently, 20 μl MTT (5 mg/ml in phosphate-buffered saline (PBS)) (Sigma, St. Louis, MO) solution was added to each well and incubated for 4 h. The formazan crystals formed by viable cells were solubilized in 150 μl dimethyl sulfoxide (Sigma, St. Louis, MO) and then the absorbance values (OD) was measured at 490 nm. Experiments were performed three times. For cytoxicity assays, cells were treated with 0, 1, 2, 4, 8, 16, or 32 µM Cisplatin (Qilu Pharmo Co. Ltd, China) (0.5 mg/ml). Each experiment was performed in triplicate. Experiments were performed three times.

### EdU incorporation

For EdU incorporation assay, proliferating NSCLC cells were examined using the Cell-Light EdU Apollo 488 or 567 In Vitro Imaging Kit (RiboBio) according to the manufacturer’s protocol. Briefly, after incubation with 10 μM EdU for 2 h, NSCLC cells were fixed with 4% paraformaldehyde, permeabilized in 0.3% Triton X-100, and stained for EdU. Then, 5 μg/ml of 4',6-diamidino-2-phenylindole was used to stain cell nuclei for 10 min. The number of Edu-positive cells was counted under a fluorescent microscope in five random fields. All assays were independently performed in three times.

### In vitro cell migration and invasion assays

For cell migration assays, 1 × 10^5^ cells in 100 µl DMEM medium without FCS were seeded on a fibronectin-coated polycarbonate membrane insert in a transwell apparatus (Costar, MA). In the lower chamber, 600 µl DMEM with 10% FCS was added as chemoattractant. After the cells were incubated for 16 h at 37 ℃ in a 5% CO_2_ atmosphere, the insert was washed with PBS, and cells on the top surface of the insert were removed with a cotton swab. Cells adhering to the lower surface were fixed with methanol, stained with Giemsa solution, and counted under a microscope in five predetermined fields (×200). All assays were independently repeated three times. For the cell invasion assay, the procedure was similar to the cell migration assay, except that the transwell membranes were precoated with 24 µg/µl Matrigel (R&D Systems, USA).

### Colony formation assay and cell cycle analysis

For colony formation assay, NSCLC cells were seeded in 6-well culture plates at a density of 100 cells/well and each group had 2 wells. After incubation for 14 days at 37 °C, colonies were washed twice with PBS and stained with hematoxylin solution. The colonies composed of more than 50 cells in a well were counted under a microscope. For cell cycle analysis, a total of 5 × 10^6^ NSCLC cells after incubation for 48 h were harvested and then washed with cold PBS. Further, cells were fixed with 70% ice-cold ethanol at 4 °C overnight. After incubation with PBS containing 10 mg/ml propidium iodide and 0.5 mg/ml RNase A for 15 min at 37 °C, fixed cells were washed with cold PBS three times. FACS caliber flow cytometry (BD Biosciences) was used to gain the DNA content of labeled cells. All the experiments were at least repeated three times.

### In vivo tumorigenesis and metastasis assays in nude mice

For in vivo tumorigenesis, a total of 1 × 10^6^ logarithmically growing A549, pc-9, SPCA-1, and H1975 cells overexpressing miR-374a or control cells were respectively subcutaneously injected in 0.1 ml RPMI-1640 medium into the left or right flank of 4–6-week-old male BALB/c nu/nu mice (*N* = 5). For the in vivo metastasis assay, 50 μl of A549, pc-9, SPCA-1, or H1975 cells (5 × 10^6^) stably expressing GFP/ miR-374a or an equal number of control cells were injected under the liver capsule of each mouse (5 mice for each group), and then carefully pushed back into the abdominal cavity after cleaning and lightly pressing the pinhole with alcohol cotton balls for 2 min. All mice were killed 4 weeks later and lungs subjected to fluorescent image detection using LT-9MACIMSYSPLUS whole-body imaging system (Lighttools Research, Encintas, CA, USA). To establish an NSCLC mouse model to test drug sensitivity, 6 × 10^5^ A549 and pc-9 or SPCA-1 and H1975 cells overexpressing miR-374a were intraperitoneal injected in 0.2 ml buffered saline into mice and tumors were allowed to grow for 3 days. Mice were then randomized into four groups for treatment of either normal saline (NS) or DDP injected intraperitoneally every 3 days. Body weights and survival of nude mice were measured regularly. Mice were maintained in a barrier facility on HEPA-filtered racks and fed with an autoclaved laboratory rodent diet. All animal studies were conducted in accordance with the principles and procedures outlined in Southern Medical University Guide for the Care and Use of Animals.

### Immunohistochemical staining

Paraffin sections prepared from in vivo experiments were used for immunohistochemistry to detect protein expression levels of CCND1 and PTEN. The indirect streptavidin-peroxidase method was utilized based on the manufacturer’s instructions. Stained tissue sections were examined separately by two pathologists. The antibodies used were rabbit anti-CCND1 (1: 250, Abcam) and anti-PTEN (1: 250, Cell Signaling Technology, Danvers, MA, USA).

### Luciferase reporter assay

CCND1 and PTEN were predicted to be the directly regulated targets of miR-374a by TargetScan (Prediction of microRNA targets) software. Fragments (452 or 350 bp) of CCND1 or PTEN 3′UTR were amplified by PCR primers (Supplementary Table 4) and cloned into psiCHECK-2 vectors (named wt). Site-directed mutagenesis of the miR-374a binding site in CCND1 and PTEN 3′UTRs was performed using GeneTailor Site-Directed Mutagenesis System (Invitrogen; named mt). For reporter assays, wild-type (wt), mutant (mt), or control psiCHECK-2 vectors were respectively cotransfected into A549, pc-9, SPCA-1, and H1975 cells together with miR-374a mimics or inhibitors. Luciferase activity was measured 48 h after transfection using the Dual-Luciferase Reporter Assay System (Promega Corporation, Madison, WI, USA). To generate a miR-374a promoter vector, a 738 bp fragment containing the two binding sites of c-JUN was PCR amplified and inserted into a pGL3-enhancer luciferase reporter vector. In addition, c-JUN mutated binding site vectors were constructed. These pGL3-enhancer-derived vector and c-JUN-expressing vectors were cotransfected into A549 or pc-9 cells and SPCA-1 or H1975 cells using Lipofectamine 2000 Reagent (Invitrogen). Luciferase activities were assayed as the aforementioned methods. Primer sequences used for PCR amplification of plasmid construction are listed in Supplementary Table S4.

### Chromatin immunoprecipitation assay

DNA–protein complexes were immunoprecipitated from A549, pc-9, SPCA-1, and H1975 cells by using the ChIP Kit (Millipore, Billerica, MA, USA) according to the manufacturer’s protocol with the following polyclonal antibodies: anti-c-JUN and normal mouse IgG (Millipore). The latter served as a control for nonspecific DNA binding. Precipitated DNA was subjected to qPCR analysis using specific primers (Supplementary Table 5) which amplified the miR-374a promoter region.

### Statistical analysis

All quantified data represented an average of at least triplicate samples. IBM SPSS v20.0 (IBM Corporation, Armonk, NY, USA) and GraphPad Prism v5.0 (GraphPad Software, Inc., La Jolla, CA, USA) software were used for statistical analysis. Data are presented as mean ± SD. One-way analysis of variance or two-tailed Student’s *t-*test was used for comparisons between groups. Fischer’s or χ^2^ test was used to identify differences between categorical variables. Partial correlations were applied in multivariate correlations analyses. Survival analysis was performed using Kaplan–Meier method. Differences were considered statistically significant when *P* < 0.05.

## Electronic supplementary material

Supplementary material

Supplementary Figure Legends
